This article has been retracted.

# Mesons from Laser-Induced Processes in Ultra-Dense Hydrogen H(0)

**DOI:** 10.1371/journal.pone.0169895

**Published:** 2017-01-12

**Authors:** Leif Holmlid

**Affiliations:** Department of Chemistry and Molecular Biology, University of Gothenburg, Göteborg, Sweden; Universitat Zurich, SWITZERLAND

## Abstract

Large signals of charged light mesons are observed in the laser-induced particle flux from ultra-dense hydrogen H(0) layers. The mesons are formed in such layers on metal surfaces using < 200 mJ laser pulse-energy. The time variation of the signal to metal foil collectors and the magnetic deflection to a movable pin collector are now studied. Relativistic charged particles with velocity up to 500 MeV u^-1^ thus 0.75 *c* are observed. Characteristic decay time constants for meson decay are observed, for charged and neutral kaons and also for charged pions. Magnetic deflections agree with charged pions and kaons. Theoretical predictions of the decay chains from kaons to muons in the particle beam agree with the results. Muons are detected separately by standard scintillation detectors in laser-induced processes in ultra-dense hydrogen H(0) as published previously. The muons formed do not decay appreciably within the flight distances used here. Most of the laser-ejected particle flux with MeV energy is not deflected by the magnetic fields and is thus neutral, either being neutral kaons or the ultra-dense H_*N*_(0) precursor clusters. Photons give only a minor part of the detected signals. PACS: 67.63.Gh, 14.40.-n, 79.20.Ds, 52.57.-z.

## Introduction

Emission of muons by spontaneous and laser-induced processes in ultra-dense deuterium D(0) [1,2] was recently reported from our group [3,4,5]. Ultra-dense protium p(0) [2,6] is quite similar in its properties to ultra-dense deuterium D(0). Both types of H(0) exist in a few different forms with different bond distances and densities. They may all be characterized as spin-based Rydberg Matter (RM) [2]. This model is based on a theoretical description by J.E. Hirsch [7]. The typical inter-nuclear distance is 2.3 ± 0.1 pm as found for D(0) in *s* = 2 in several studies [1,8,9]. This corresponds to a density of 10^29^ cm^-3^ or >100 kg cm^-3^. This density is a factor of 10^5^ higher than in ordinary condensed hydrogen. Recently, much more precise inter-nuclear distance measurements have been done by rotational spectroscopy, giving distances in D(0) with a precision of ±0.003 pm [10]. MeV particles are ejected by laser-induced processes in both D(0) and p(0) [11–13]. Also, normal D+D fusion processes giving ^4^He and ^3^He ions were shown to be initiated by a relatively weak pulsed laser [14]. Laser-induced nuclear fusion in D(0) gives heat above break-even, as reported in Ref. [15]. Recent studies show that the MeV particles ejected from H(0) decay within 100 ns [16–18].

The present study employs a combination of magnetic deflection and time (time-of-flight, TOF) measurement methods to identify the ejected MeV particles. Large fluxes of particles with velocities 10–20 MeV u^-1^ [11–13] definitely indicate nuclear reaction processes. However, ordinary D+D fusion reactions only give an energy up to 3.0 MeV u^-1^ in the first reaction step, and up to 14.7 MeV u^-1^ in the second step of the reactions. Thus, other nuclear processes take place. The ejected mass is here found by magnetic deflection to be less than unity but much larger than the electron mass. At least two different masses are observed, which agrees with the particles being light mesons. The particle decay times observed agree very well with this conclusion.

In general, a mix of mesons mainly kaons and pions, giving muons, is observed. Both neutral and charged mesons are formed, which means that time measuring methods are preferred here instead of electric analyzing fields [19,20]. Further, without the time measurements, the very important particle decay time information would be lost. Two-collector and three-collector experiments in the same system have been published previously [16,21–23]. At short distance, such experiments indicate that a particle transport delay exists between the collectors, corresponding to the particle distance travelled, thus proving that massive non-relativistic particles are observed. The particle velocity observed is normally at 10–20 MeV u^-1^ at the peak of the distribution, thus up to *v*_*p*_ = 0.2*c*. However, when the distance to the second (outer) collector is increased, this picture changes to give a too short TOF and a too high signal at the outer collector as in Refs. [15,17,23]. The particles then move with a velocity close to the speed of light *c* and the TOF distribution is sharper at long distance [17]. This indicates that some particles in the beam decay during the flight, and this TOF distribution sharpening effect (and the simultaneous increase in signal intensity) also shows that the signal is not due to photons. Thus, the particles change their velocity and also their mass during the flight in the beam.

Results on ultra-dense hydrogen from other groups exist. A superconductive hydrogen state consisting of very high-density hydrogen clusters in voids (Schottky defects) in palladium crystals has been studied experimentally by Lipson et al. [24]. This effect was attributed to Bose-Einstein condensation [25] or a Casimir effect [26]. Such ultra-dense hydrogen clusters may give increased fusion gains from suitably prepared targets [27]. The close relation between these hydrogen clusters and ultra-dense hydrogen H(0) has been pointed out [28].

Related results on laser-induced nuclear processes exist. Such studies mainly aim at ignition of nuclear fusion by ICF (inertial confinement fusion), for example by initial laser compression of a hydrogen fuel target to high pressure and temperature. This possibility was proposed already in the 1980's [29]. A similar compression method is used with the "world's most powerful laser" at the National Ignition Facility (NIF) in the US [30]. The amount of fusion is there measured by the neutrons released. Thus, other processes than normal D+T fusion are not investigated. The progress in such inertial-confinement fusion (ICF) studies is plagued by instabilities in the compressed hydrogen fusion fuel [31]. ICF schemes using lower compression and a fast igniting laser pulse are also under development [32]. On a smaller scale, interesting reports on laser-induced fusion reactions in hydrogen clusters exist [33,34]. In laser-induced fusion reactions using a 10 TW laser [35] the neutron energy was found to be up to 4 MeV. This was suggested to be due to deuteron acceleration in the laser-produced plasma.

Related results also on the laser-induced formation of MeV particles from hydrogen exist. Multi-MeV particles, mainly protons, were formed in an experiment with a 2 J, 30 fs laser at various targets [36]. The high particle energy was suggested to be due to the plasma formed. In another case, a 1–2 MeV mono-energetic proton beam was obtained from a hydrogen gas jet by using a 1 TW CO_2_ laser [37]. There exists also one report on the formation of alpha particles at MeV energy during hydrogen desorption from a complex solid phase containing Pd [38]. This solid phase may act as a hydrogen active catalyst. Mesons have been produced in large facilities by laser-derived scattered photons at GeV energy, like p + γ giving K^+^ and π^+^ among others [39]. Mesons can also be formed by fast protons from fusion reactions like p + d, for example giving ^3^He and K^+^ + K^-^ [40].

## Theoretical background

Ultra-dense hydrogen H(0) is the lowest energy form of hydrogen atoms. This material was previously named H(-1) since it was thought to be an inverted form of matter where nuclei and electrons had exchanged their roles. Since it now is clear that the description of H(0) as a spin-based form of Rydberg matter [2] agrees well with experimental results, the angular momentum is now used as the characteristic parameter as for other types of Rydberg matter [41]. Several forms exist, but the most common form has a H-H bond distance of 2.3 ± 0.1 pm [1,8,9]. H(0) is closely related to dense hydrogen H(1) which has an H-H distance of 150 pm. More background is given in a recent review on Rydberg matter [41]. The relations in energy and distances are also shown in Fig 1. The microscopic structure of H(0) is given by chain clusters H_2*N*_ with *N* integer. Such clusters contain pairs of nuclei which rotate around the axis in the cluster [10,42]. The ultra-dense materials are quantum materials with properties like superfluidity and superconductivity [43]. These properties were verified for D(0) by a fountain effect [44] and a Meissner effect for both D(0) [45] and p(0) [46], both observed at room temperature. The superfluid nature of both D(0) and p(0) is directly observed in experiments which use this property to form thin moving liquid films on metal surfaces [6,47]. It is found that condensation to D(0) does not take place on organic and inorganic polymer surfaces [13,48]. The similarity of D(0) to other superfluids was first discussed by Winterberg [49,50].

**Fig 1:** Relation between ultra-dense hydrogen H(0) and other forms of hydrogen. The blue arrow indicates the real-time switching between the two forms H(1) and H(0). The axes are not to scale.

The theory for the time-of-flight experimental proof of the extremely short bond distances in H(0) is summarized here. Recently, an even better method was used to observed the bond distances for spin quantum number *s* = 2, 3 and 4 in D(0), namely rotational emission spectroscopy [10]. The precision of such measurements turns out to be very high, around ±0.003 pm from a large number of rotational lines. When a chemical bond is broken by photons for example by a relatively weak laser beam as used here, the electrons in the bond are either excited to higher energies (orbitals) or are ejected from the bond, leaving one or several ions behind. The excess energy given to the ionic fragments depends on their distance when they are formed by the electron removal. If this excess energy is larger than the bond energy to other atoms in the material, the ion (atomic or molecular) may be ejected from the material. This process is a form of Coulomb explosion (CE). The maximum energy release is easily calculated from the initial distance between the charges when they are formed (thus when the electrons are removed). Thus, it is possible to determine the initial repulsion energy between the ions by measuring the kinetic energy of the fragments at a large enough distance. The distance between the ions before the break-up is found directly from the Coulomb formula as

$$r=\frac{1}{4\pi \varepsilon_{0}}\frac{e^{2}}{E_{kin}}$$

where *ε*_0_ is the vacuum permittivity, *e* the unit charge and *E*_*kin*_ the sum kinetic energy for the two fragments (KER) from the CE. The fraction of the KER that is observed on each fragment depends of course on the mass ratio of the fragments. The kinetic energy is determined most easily by measuring the TOF of the particles and converting this quantity to kinetic energy. This requires that the mass of the particle is known or can be inferred, which is relatively easy in the case of hydrogen. Now, the normal kinetic energy (velocity) from laser-induced CE determined by time-of-flight in numerous experiments is 315 eV u^-1^ [1,8,9]. The fastest particles observed when working with deuterium have reasonably a mass of 2, thus a kinetic energy of 630 eV. This means an initial distance of 2.3 pm between the ions. This distance is a few percent of a normal chemical bond, which means that (100/2.3)^3^ = 8×10^4^ gives the order of the density of this ultra-dense material relative to ordinary materials, or a density of the order of 100 tons per dm^3^. It should be observed that the energy of the fragments generated by the CE does not change with the laser intensity. This means that any acceleration of the ions due to the laser is excluded, which is also clear from the relatively low laser intensity used.

The origin of the particle signals observed here is clearly laser-induced nuclear processes in H(0). The first step is the laser-induced transfer of the H_2_(0) pairs in the ultra-dense material H(0) from excitation state *s* = 2 (with 2.3 pm H-H distance) to *s* = 1 (at 0.56 pm H-H distance) [2]. The state *s* = 1 may lead to a fast nuclear reaction. It is suggested that this involves two nucleons, probably two protons. The first particles formed and observed [16,17] are kaons, both neutral and charged, and also pions. From the six quarks in the two protons, three kaons can be formed in the interaction. Two protons correspond to a mass of 1.88 GeV while three kaons correspond to 1.49 GeV. Thus, the transition 2 p → 3 K is downhill in internal energy and releases 390 MeV. If pions are formed directly, the energy release may be even larger. The kaons formed decay normally in various processes to charged pions and muons. In the present experiments, the decay of kaons and pions is observed directly normally through their decay to muons, while the muons leave the chamber before they decay due to their easier penetration and much longer lifetime.

The observed collector signal in the experiments described here is often due to a fast intermediate particle M which is formed and decays like A → M → N. Thus, largely the same time dependence is observed by collectors at short and long distances, if the particle velocity is high. This general conclusion is modified by the transverse energy given by the decay processes to the products, which means that some particles do not reach the outer collector. The time dependence of the signal M is easily derived from the rate equations [16,17] for $\text{A}\overset{k_{1}}{\to }\text{M}\overset{k_{2}}{\to }\text{N}$

$$-\frac{dn_{\text{A}}}{dt}=k_{1}n_{\text{A}}$$ (1)

$$\frac{dn_{\text{M}}}{dt}=k_{1}n_{\text{A}}-k_{2}n_{\text{M}}$$ (2)

as

$$n_{\text{M}}=\frac{k_{1}}{k_{2}-k_{1}}n_{\text{A}}{}_{0}(e^{-k_{1}t}-e^{-k_{2}t})$$ (3)

Time constants τ = 1/*k* are used in the experimental results below. It should be realized that this type of interpretation implies that the particle transport time from the target is short and relatively constant for all particles and that the width of the apparent TOF distribution is mainly due to the particle creation and decay processes. This indicates a transport time that is considerably shorter than the other time constants. A decay chain can also contain more intermediates. The formulas for two intermediates are quite straightforward and have also been tested, but with no large improvement.

The time variation of the signal at the collectors needs some further consideration. With a decaying particle ejected from the laser target, a few limiting situations can be understood. If the particle velocity is high thus the decay takes place outside the detecting collector, the signal at the collector will only vary with the rate of emission from the target. If on the other hand the velocity of the particles is very low, all the particles will decay before they reach the collector. In such a case, the particles ejected from the decay at the target will be observed by the collector. This means that the signal time development follows the decay time of the decaying particles. In the intermediate case where the decay time is of approximately the same size as the time of transport to the collector, the signal at the collector will be distorted and shortened relative to the true decay at the collector. If there are two intermediates in a decay chain a similar situation exists since the decays all start at zero time. A decay chain $\text{A}\overset{k_{1}}{\to }\text{M}\overset{k_{2}}{\to }\text{N}\overset{k_{3}}{\to }\text{O}$ implies that the N particles are converted to O as soon as they are formed which is at zero time. Of course, a typical signal decay of N may require that both A and M are exhausted, so the total time before N decays is longer when the chain starts from A than if the chain started from M. Thus, more complex time variations than a simple exponential may indicate that two intermediates exist and decay in the beam.

The mesons that exist in the flux from the target have short lifetimes and decay with different energies which give large kinetic energy to the particles formed. This means that most particles formed in the beam will receive kinetic energy in another direction than the beam direction, and they may not be able to stay in the beam and reach the collectors if not their initial velocity before decay already is very large. This also means that the spatial distributions for different particle types are likely to be slightly different. However, there exist some meson decay processes which form only one meson or muon, and light leptons otherwise. These processes are

$${\text{K}}_{\text{L}}^{0}\to \pi^{+}+e^{-}+\nu_{e}\;with\;\tau =52\;ns$$ (4)

$${\text{K}}^{+}\to \mu^{+}+\nu_{\mu }\;with\;\tau =12\;ns$$ (5)

$$\pi^{+}\to \mu^{+}+\nu_{\mu }\;with\;\tau =26\;ns$$ (6)

and their negatively charged counterparts. The probabilities of these decay branches are 39%, 64% and 100% respectively [51]. The light leptons will remove most of the excess energy, leaving the heavy particle from the decay still in the beam direction with largely unchanged kinetic energy. Since the muons are less easily observed at the collectors then the mesons, the decay to a muon may be observed as a disappearing pion or kaon, like particle M in Eq (3).

In the experiments, also relativistic particles are observed which appear to have a decay time of 13–16 ns. These particles are thus apparently fast K^±^. The most likely formation process is directly from the initial stationary H_*N*_(0) species on the target surface which undergo an internal nuclear process to kaons.

Also, a time constant close to 40 ns is often observed in the experiments. It is closely related to the two time constants at 26 and 13 ns. If these two time constants exist in a chain, preferentially with the time constant 26 ns last, the result may be an apparent 39 ns time constant. There exist two charged kaon decay processes which may give this behavior, namely

$$\begin{array}{l} {\text{K}}^{+}\to \pi^{+}+\pi^{0}\\ \text{or}\to \pi^{+}+\pi^{+}+\pi^{-} \end{array}$$

with 12 ns time constant, normally at 21 and 6% probability [51]. They will both then give charged pion decay with 26 ns time constant. In this way the two time constants are combined as required. Both these processes are very energetic and it may not always be possible to observe the pion decay from them since the particles may leave the beam. This agrees with the results below.

## Experimental

A Nd:YAG laser with pulse energy of < 0.2 J was used, with 5 ns pulses at 532 nm and 10 Hz repetition rate. The source used for producing D(0) and p(0) is described in the literature [8]. In the source, a potassium doped iron oxide catalyst sample [52,53] forms D(0) from deuterium gas (99.8% D_2_) or p(0) from H_2_ gas ((99.9995% pure hydrogen, naturally containing only 0.016% D). The ultra-dense material formed falls down to the target plate below the source where the laser beam impinges. The direction of the flux from the target to the collectors is at approximately 60° towards the normal of the target and at 45° relative to the impinging laser beam. The set-up used is shown schematically in two forms in Fig 2 [1,12]. The vacuum chamber has a base pressure < 1×10^−6^ mbar. The collector part is pumped separately. The D_2_ or H_2_ gas pressure admitted to the chamber is up to 1×10^−5^ mbar (uncorrected ionization gauge reading). In several experiments, the target was Ni foil with a Pt rod spot welded on it. The foil was mounted with a 45° slope towards the vertical. The laser beam is focused on the foil with an *f* = 400 mm spherical lens. The intensity in the beam waist of (nominally) 30 μm diameter is relatively low, ≤ 3×10^12^ W cm^-2^ as calculated for a Gaussian beam. The foil collectors used in the time measuring experiments consist of 1–3 layers of 20 μm Al foil on a steel ring, specified more exactly in the text where needed.

**Fig 2:** Horizontal cut through two layouts of the apparatus, with various parts indicated. The upper form is for most time measuring experiments, the lower one for the magnet deflection experiments. The inner pin collector is at 64 cm distance from the target. It is a 1 mm diameter pin which is mounted on a rotatable flange. The offset on this flange is 26 mm so deflections ± 20 mm are detectable. The outer collector is at 163 cm from the target.

In the wall of the cylindrical chamber in Fig 2, an aperture with diameter 5 mm limits the angular spread of the particle flux to the collectors. The flux in the beam is in some of the experiments analyzed by a magnetic field provided by two or four small permanent rectangular magnets (ferrite Y28 magnets with length 30 mm, width 10 mm and height 5 mm, remanence 400 mT) above and below the beam to the collectors. The magnets were mounted on an arm which could bring them in and out from the beam to the collectors. The distance between the (inner) pole faces was 5 mm. The magnetic field strength has been measured with a Hall effect sensor (Allegro A1326 giving 2.5 mV G^-1^). The field strength between two magnets in the beam was 100 mT, while it was 160 mT using four magnets in pairs above and below the beam. Just behind the magnets, a central opening of 4×4 mm on the arm was used to define the beam. Further in the beam direction at 2 cm distance, a beam defining slit with width 0.8 mm and vertical height 5 mm was mounted in the wall between the central chamber and the separately pumped collector chamber, at 22 cm distance from the target. The magnets have a width perpendicular to the beam of 10 mm with a distance between the pole surfaces of 5 mm. Thus the variation in field strength over the effective slit width of considerably less than 0.8 mm is negligible. The first (inner) collector in the magnet experiments was in the form of a vertical pin of 50 mm length and 1 mm diameter which could be moved sideways by rotating the flange on which it was mounted with an offset as shown in Fig 2. The distance of this pin collector from the target was 64 cm. A laser pointer on the same flange was used to observe the rotation of the flange and thus the sideways motion of the pin. The step size used in the deflection measurements is 0.63 mm, smaller than the pin diameter. No large signal was observed outside ± 3 mm sideways motion relative to the central beam. The pin current (and the other collector signals) is measured directly with a 300 MHz digital oscilloscope with a 50 Ω coaxial input (Tektronix TDS3032 with rise-time of 1.2 ns). The bias on the pin is zero or -24 V. The typical signal is in the mA range, with the current density at the inner collector of the order of 25 mA cm^-2^. With negative bias, no secondary electrons due to photons from the target can reach the pin. A diode at the laser gives the trigger signal. The length of the cabling is adjusted so that the maximum zero point error in the trigger signal is 3 ns at the oscilloscope. A signal delay of 1–2 ns exists with negative bias. The laser pulse width is 5 ns, which means that a precision much better than half this value (half-width of the peak) thus 2–3 ns is not meaningful. The oscilloscope rise time of 1.2 ns will not give any substantial broadening of the signals in time.

Checks with magnets outside the chamber show no electrons in the beam to the collectors. Of course, low energy electrons giving the positive collector signals are released at the collectors by the impinging particles independent of their polarity. These currents are influenced by strong external magnets as expected. Neutron emission was monitored by using bubble detectors (Bubble Technology Industries, BTI) types BN-PND for high energy (<15 MeV) and BDT for thermal neutrons. They were located outside the vacuum wall of the chamber. Typically no bubbles are formed during the experimental runs.

The procedure used in the determination of fits to the experimental data differs from many cases of radioactive measurements. This is due to the fact that the signal observed is not a particle count but a voltage signal observed with an oscilloscope. The digital oscilloscope gives a recorded signal of the voltage at each measuring point, spaced 0.2 ns apart. The voltage value observed is of the order of 100 mV, thus with a signal current of 2 mA. This corresponds to a number of particles observed per time bin of 0.2 ns of 2.5×10^6^. Each time spectrum in most of the figures contains thus 2.5×10^9^ particles in the 1000 time bins shown in the figures. The treatment of the results here is as normally used for analog (continuous) results but not normally found in radioactivity measurements, by determining model parameters by least-squares non-linear fits, as described further below. It is thus not possible to use a simple test like chi-square to estimate the probability of the fits between theory and experimental results. Typical result for a truly excellent 1% fit in each point with 10^6^ particles would be χ^2^ = 10^8^/10^6^ per bin (point), thus total χ^2^ = 10^5^ for 1000 bins or degrees of freedom. This will be rejected due to too large variation. To have a statistically acceptable value of χ^2^ = 10^3^ for 1000 bins or degrees of freedom requires a 0.1% fit in each point, thus better than the precision and accuracy of most measuring instruments. Thus, such values are not obtainable. Below, the lifetime for pions is determined from the fits within 1% of the correct value, which indicates that the procedure used is not only the best for analog results but also that it gives correct physical results.

## Results

### Energy spectroscopy of laser-induced particles

Experiments that identify the laser-induced particles by scintillator-based energy spectroscopy have been done in another closely located apparatus in the laboratory [4,5]. Such results are included here to give direct evidence with another method that muons are indeed formed by the laser-induced processes. The processes that give muons are both laser-induced [5] and spontaneous [3]. A typical experiment is shown in Fig 3, where both a plastic scintillator (PS) and an Al metal converter [4] are used to detect the muons and other particles from the laser-induced nuclear processes in the D(0) layer on the target. At channel No. below 200, the beta-like electron distribution initiated by muon decay and negative muon capture in the Al converter (and in the glass in the photo multiplier) is observed. At channel No. 200–500, the muon and background particle signal from the PS is observed. At channel No. > 600, MeV particles (positive muons) giving photons in the PS are observed. Further results are given in Refs. [3–5]. Muons are thus regularly detected in the laser-induced experiments.

**Fig 3:** Many-channel analysis (MCA) energy spectrum using a plastic scintillator and Al converter [4] in a small chamber with D(0) generation on the laser target. See further text.

### Two-collector time measurements

Time measurements using two and three collectors in line to analyze the laser-induced flux from H(0) have been published [16,17,21–23]. In Fig 4 such results are shown with the present setup with large foil collectors as in the upper sketch in Fig 2. The geometry of the setup is such that almost all particle flux to the inner collector also reaches the outer collector, assuming a point source at the laser target and linear propagation. In Fig 4 the signal is described by an intermediate decaying particle flux following Eq (3). It should be realized that this type of interpretation implies that the particle transport time from the target is short and that the width of the distribution is mainly due to the particle creation and decay processes. The overall shift of the signal rise thus the transport time between the collectors is close to that due to the velocity of light (4 ns for 0.99 m). However, the signal decay to the inner collector is considerably slower than that to the outer collector, with a decay time constant of 20 ns instead of 13 ns to the outer collector. Thus, some slower particle flux may have been lost between the collectors.

**Fig 4:** Two-collector experiment with p(0) on a Pt target surface. Negative collector bias.

A similar case is shown in Fig 5. In the log plots used there, the good agreement with the intermediate decaying particle formula Eq (3) is seen better. The inner collector signal has a decay time of 28 ns, while the outer collector has a decay time of very accurately 13 ns. Assuming that the signal decay is due to a decay to muons which then give the collector signal, the inner collector signal could be due to pions with 26 ns decay time constant at rest, while the outer collector signal could be due to charged kaons with 12.4 ns decay time constant. The signal from decay of charged kaons at the inner collector is smaller than that from the pions and thus not clearly observed there, as seen directly in Fig 5. The reason why the pions are not clearly observed at the outer collector is probably that they have a large transverse kinetic energy from their formation which brings them out from the beam to the outer collector. The inner collector signal may in fact be a little more complex, containing two different signal distributions as described further below.

**Fig 5:** Two-collector experiment with D(0) on a Ta target surface. Negative collector bias.

### Relativistic charged particles

Time measurements with and without magnet deflection show that very fast particles exist in the laser-induced flux from the target with H(0) coverage. The measurements involve comparisons between the signals with and without a deflecting magnetic field in the beam. In Fig 6, the direct difference signals are shown for the signal to the outer collector with zero and negative bias. No scaling is used but only a direct subtraction since only the magnet position is changed. The material used here is p(0) but D(0) gives similar results. Also the signal at the inner pin collector is similar, as shown in Fig 7. The difference signal is thus due to charged particles of positive or negative sign which have been deflected more than 5 mm at the outer collector (with width 10 mm in these experiments) so they miss this collector. The deflected part of the signal is displayed, with an analysis in the form of an intermediate particle. It is seen directly that the signal at the outer collector is larger than that at the inner collector. This is expected from the small slit used to define the beam: since the inner pin collector in this experiment is only 1 mm wide, part of the flux to the outer collector passes the inner collector. It is also seen directly in the figures that the difference signal is faster at the peak than the other signals. Thus, the difference signal is not due to shadowing by the magnet holder or any similar artifact. An experiment always starts by optimizing the laser beam position on the target, by maximizing the signal at the outer collector. This type of experiment has been performed numerous times with different laser optimization and with similar results. With a weaker magnetic field than used for the figures shown, the deflected (difference) signal is generally smaller.

**Fig 6:** Magnet deflection experiment at outer collector at 163 cm distance. Signal with no magnet and difference signal (no magnet—magnet) are shown. The difference signal is fit by the intermediate particle with data shown. p(0) on Pt target surface. Magnetic field strength 0.16 T.

**Fig 7:** Magnet deflection experiment at inner pin collector at 64 cm distance. Signal with no magnet and difference signal (no magnet—magnet) are shown. The difference signal is fit by the intermediate particle with data shown. p(0) on Pt target surface. Magnetic field strength 0.16 T.

The charged particle signal rise time of 2 ns with zero collector bias is close to the rise time of the oscilloscope. Thus the real rise time of the signal is considerably faster (close to 1.6 ns) and slightly faster than the laser-pulse rise time (5 ns broad laser pulse). The use of negative bias on the collector is seen to give a further delay of 1–2 ns, but it is otherwise consistent with the results with no bias. The transport time between the two collectors is directly found as the difference between the start times or the peak times of the signal at the inner and outer collectors. Since the same cable is used to sequentially connect one or the other of the collectors to the oscilloscope, this means that all other factors cancel out in the measurement. The time found between the collectors is 2.5–4 ns for the various examples. The time for light to move the 990 mm between the collectors is 3.3 ns, in close agreement with these observed charged particle TOFs. Thus, the charged particles observed have close to relativistic velocities.

The deflection at the outer collector can be calculated for various velocities of particles with different mass. The results are displayed in Fig 8, showing the limiting mass which is just deflected outside the collector and the dark part of the plot where the lost particles exist. Thus all particles with the same velocity but less than this limiting mass are deflected outside the collector. The deflection results indicate mesons, probably charged kaons and pions, as the particles deflected. Leptons like muons may also be possible, but lighter leptons like electrons are deflected by the geomagnetic field and cannot reach the outer collector. The decay times observed of 13–16 ns agree with charged kaons. Thus the relativistic particles observed are probably charged kaons. The observed decay time of 16 ns relative to the value 12.4 ns at rest corresponds to a velocity of 0.64*c* or 280 MeV u^-1^.

**Fig 8:** Calculated particle mass and velocity giving deflections of 5 mm at the outer collector with an 0.16 T deflecting magnetic field in Fig 6. The shaded area indicates particles deflected outside 5 mm. The particle energies used for the calculated points from left to right are 10, 20, 50, 100, 200, 500 MeV u^-1^ and 1 GeV u^-1^.

### Particle separation by metal foils

Some of the particles ejected from the laser target at high energy penetrate easily through metal foils. This has been reported previously [11,12,54]. A very clear case is shown in Fig 9 where the inner collector (beam flag) is a thin steel ring with just one 20 μm thick Al foil covering the opening. It is almost impossible for any particles to scatter around its edge (another metal plate ring reaching to the wall prevents that). The signal to the outer collector at 1.6 m distance from the target is shown, with the inner collector open and closed. The signal is interpreted as an intermediate particle in both cases. The outer collector signal with the foil flag closed is smaller, about 30% of the peak intensity, and seems to be delayed approximately 3 ns. However, by subtracting the "closed" signal from the "open" signal, a much smoother curve shape for the outer collector signal is obtained as seen in the upper panel in Fig 10. This indicates that the penetrating ("closed") signal is a slightly slower type of particle which penetrates through the Al foil without intensity loss. The smooth difference curve at the outer collector still does not seem to correspond to just one process, but at least two different signal contributions combine in this signal. However, the main peak is well fit by a simple intermediate with 15 ns decay time. By subtracting the “closed” outer collector signal also from the signal to the inner collector (with multiplier equal to 2 since the angular coverage of the inner collector is larger than for the outer collector in this case), it is possible to match the peak of the resulting curve well with the same decay time-constant as for the outer collector difference (15 ns, charged kaon decay). This indicates that the "closed" signal is due to a special particle, probably a neutral particle since it can penetrate so easily through the Al foil. The oscillations in the outer collector signals indicate a boson giving lepton pair formation and charge oscillations [16]. Thus the penetrating signal is likely due to a long-lived neutral kaon ${\text{K}}_{L}^{0}$ with decay time 52 ns. The apparent shorter decay time in the "closed" signal may be caused by a relatively low velocity of the neutral particles and partial decay of the kaons before they reach the outer collector. This agrees with the slower peak of this signal, as seen in Fig 9. Another possible process is the regeneration of the shortlived ${\text{K}}_{S}^{0}$ type of kaon by the passage through the metal foil [55].

**Fig 9:** Effect of the Al foil filter. The inner collector is a 20 μm thick Al foil on a wire frame. D(0) on a Pt target. Collector signals with interpretations as intermediate particles with data shown.

**Fig 10:** Removal of the neutral penetrating particles in Fig 9, giving smoother, more easily interpreted signals. The decay times at both collectors become the same. See text.

### Intermediate decaying particles

A more complex behavior can be seen by using experimental conditions that give several different signal parts at the collectors. Typical examples are shown in Figs 11 and 12 for the inner and outer collector signals with bias 0 and -24 V. The different parts seen in the figures have been matched by the intermediate particle formula in Eq (3). The parameters found are collected in Table 1. This is not a full modeling of the entire curves, since the overlaps of the different parts are difficult to include, thus only the parameters for each separate part of the curves are given. An interpretation of the various peaks is also given in Table 1. The first fast peaks are due to very fast particles from the target with short decay, probably shorter than the laser pulse. Thus, these peaks are similar to the laser pulse. The longer decay times observed in some cases in Table 1 are due to particles that decay at the target or in the beam close to the target, giving fast products that move to the collectors and are detected there. The effect of the negative bias is to accelerate away slow electrons ejected from the collectors by the impinging particles, thus increasing the positive signal observed. This gives a smoothing of the signal and a delay of the signal of 1–2 ns. The negative bias also gives apparent differences in the particle interaction with the collectors. For example at the outer collector in Table 1, a signal apparently due to charged pion decay is observed with negative bias. The pions seem to pass through the collector with much smaller interaction in the case of zero bias, giving a signal hiding under a charged kaon decay.

**Fig 11:** Two-collector experiment with D(0) on Pt with zero bias. Complete intermediate particle data in Table 1.

**Fig 12:** Two-collector experiment with D(0) on Pt with negative bias. Complete intermediate particle data in Table 1. The outer collector signal is fitted by a non-linear fit procedure with the parameter values given in the table, at convergence.

**Table 1:** Best adjusted parameters for the intermediate particle signals shown in Figs 11 and 12. D(0) on a Pt surface. Inner collector at 64 cm, outer collector at 163 cm. Time constants with error limits are found with a non-linear fit procedure (see text). The average fit in % is determined as *s*/<*x*> where *s* is the absolute difference between the signal and the model and <*x*> is the average signal.

Outer collector	Bias 0 V				Bias -24 V			
Peak size (V)	0.19		0.018				0.26	
τ_1_ (ns)	5		8				4.81±0.05	
τ_2_ (ns)	3		40				23.7±0.1	
Delay (ns)	12		24				13	
Average fit (%)	7.7 (12–25 ns)		18 (35–200 ns)				6.8 (15–200 ns)	
Inner collector	Bias 0 V				Bias -24 V			
Peak size (V)	0.85	0.23		0.04	1.05	0.82		0.21
τ_1_ (ns)	3	4		4	4	4		4
τ_2_ (ns)	1	8		52	3	8		80
Delay (ns)	9	12		12	9	12		12
Average fit (%)	12 (9–15 ns)	3.1 (15–32 ns)		2.4 (40–200 ns)	19 (9–14 ns)	3.8 (18–25 ns)		7.8 (50–200 ns)
Interpretation	Fast	Fast	Charged kaon + pion	Neutral kaon	Fast	Fast	Charged pion	Neutral kaon + more

Numerical fits of Eq (3) to the particle timing data like those in Figs 11 and 12 require non-linear fits with several adjustable parameters, since several different particles contribute to the distributions, as seen in most cases in Table 1. This presents a quite complex numerical problem due to the exponential functions which means that the parameters are strongly dependent on each other. However, in Fig 12, the signal at the outer collector is well described by just one particle type. Thus, Eq (3) can be used with three or four adjustable parameters to fit the data in this case. The standard errors for the decay time constants are given in this case in Table 1 at convergence, using the non-linear Marquardt-Levenberg fit procedure in the program SigmaPlot 13. Thus the decay time constant is found to be τ_2_ = 23.7 ± 0.1 ns. A fit of similar quality can also be found with τ_1_ = 3.46 ± 0.05 ns and τ_2_ = 26.5 ± 0.2 ns, which may be closer to the real time constant values as shown below. The standard errors given by the non-linear fit procedure are calculated for each parameter independently, and the parameters are strongly dependent as is normally the case in an exponential fit. The combined error limits which are more complex to calculate are larger. However, the good fit means that the intermediate particle model is valid.

Evaluating the single exponential slope of the signal to the outer collector in Fig 12 is more accurate. Using the time range 30–150 ns with 600 measured points gives a decay time constant of τ_2_ = 25.28 ± 0.05 ns from a two-parameter non-linear fit, while a two-parameter linear fit to the logarithm of the signal gives τ_2_ = 26.37 ± 0.05 ns. Thus the true error limit is more likely ± 0.6 ns to make these two values agree at τ_2_ = 25.8 ns. This is close (better than 1%) to the best tabulated value for charged pions at 26.033 ns [56]. This good agreement supports the interpretation of these data as due to pion decay.

In Table 1, also other measures of the goodness-of-fit are included. For each part of the curves which agrees with a set of parameters in the intermediate particle model, the average departure at each point is calculated as absolute deviation at each point (calculated between the experimental signal and the computed curve for the intermediate particle model) divided by the average of the signal over the used time range. This gives a meaningful estimate of the fit. In some cases shown this fit is quite good especially considering that often several different types of particles contribute to the signal. When an interpretation as just one type of particle is possible as in some cases in Table 1, the best fits are found.

### Decay times

A further possibility to investigate the behavior of the decaying particles is to vary the laser intensity. This will vary the conditions for the meson production but may anyway help to clarify the various decay steps. In Figs 13 and 14, the complex decay curves at the outer collector at 1.6 m distance are shown with and without a negative bias at the collector. Two meson time-constants at 13 ns (charged kaons) and 26 ns (pions) are there shown to combine to also form a time constant equal to their sum of approximately 39 ns. Since the decay steps are coupled (the kaon decay may form the pions as described in the theoretical section), the two sequential decay steps give this effect. Thus there are two intermediate particle species in this chain. This explains the 40 ns decay time constant obtained in one case in Table 1 as due to the decay of pions after their formation by decay from charged kaons. The separate time constants can also be measured with good precision. An example of the measurement of the charged kaon decay at the outer collector is shown in Fig 5, with 13 ns decay time constant.

**Fig 13:** Variation of laser pulse energy, signal at outer collector, zero bias. D(0) on Ta target surface. Combined behavior of two decay time constants at 13 and 26 ns, giving also 39 ns at long time.

**Fig 14:** Variation of laser pulse energy, signal at outer collector, negative bias. D(0) on Ta target surface. Combined behavior of two decay time constants at 13 and 26 ns, giving also 39 ns at long time.

### Magnetic deflection

To study the energy and mass of the particles observed, magnetic deflection experiments have been done at two different magnetic field strengths. To use two field strengths was necessary due to the large neutral signal and the large spread in particle velocities at 0.15–0.75 *c* or 10 MeV u^-1^–500 MeV u^-1^. The deflection of the particle flux was measured with the movable pin collector shown in Fig 2. Due to the somewhat damaging interaction between the laser beam and the target, it is not optimal to use the same laser beam spot in every experiment, since constant conditions for each of the eight different experiments of course were sought. (Due to the superfluid properties of the ultra-dense hydrogen, it is still possible to have constant conditions during each experiment since the layer on the target surface is rapidly renewed [6,44,47]). Thus, the laser beam position on the target is slightly different for different experimental runs, even if the target is also moved to find the optimum position. Another reason for this is the variation in the beam composition between experiments, with different types of particles probably having different spatial distributions in the beam due to differences in the meson decay patterns. See further in the Discussion section. However, the size of the variations is small as described here.

The measurements were started by maximizing the signal to the outer 10 mm wide collector by adjusting the laser spot position on the target, and the sideways position of the target in front of the narrow 0.8 mm wide slit in the beam to the collectors. The beam passed through the narrow slit in the central chamber wall, and the collector position was constant. The typical expanded beam width was 2.5 mm at the pin collector, as expected from a point-source at the target through the 0.8 mm width at the slit. However, small differences in the alignment exist between the experiments due to the slightly different locations of the small beam spot on the target. The collector and slit layout means a maximum sideways position of the laser spot on the target of 1.2 mm and a sideways position at the pin collector of -1.2 mm, if a narrow beam was maximally misaligned to one edge of the slit. However, the alignment procedure optimized the position of the laser spot for maximum signal transmission and thus a central location of the expanding beam relative to the narrow slit and the collector. The pin signal gave directly both the beam profile and the beam center, and the beam center was then used as the zero point for the steps of the pin collector. The data with and without the deflecting magnet were then taken directly in order for each pin step. The deflection TOF-angular distributions are consistent using the actual center of the beam, which means that adjustment factors like edges or non-alignments of other types are unlikely to influence the results using this alignment procedure. Thus, the signals and especially the difference signals are independent of the actual laser beam position on the target, and internally compatible for the results with and without the magnet in the beam since they are measured almost simultaneously with no realignment. Data from four experiments are shown here, but four further experiments with other parameter combinations (p(0) or D(0), zero or negative bias, magnet strength 0.10 or 0.16 T) exist which agree with the ones shown. The good alignment can be seen in the symmetric shape of the signal without magnet in each experiment. However, due to the large number of particle types formed, all types will not have the same distribution in the beam. See further in the Discussion section.

In all cases, deflection distributions (signal time distribution vs. pin collector location) have been measured a) both with p(0) and D(0) on the target surface, b) with negative bias and with zero bias, and c) with and without the magnet in place in the beam, inside the slit in the main chamber wall. The almost simultaneous results without and with the magnet have been subtracted to give a deflection signal for *I*(no magnet)—*a*×*I*(magnet). Such difference distributions are the ones displayed here together with the direct signal with and without magnet. The factor *a* is normally 1.2. The value 1.2 is based on the height of the two beam defining slits, with the fixed slit of 5 mm height and the movable slit (on the magnet holder) of 4 mm height. The exact value of the *a* factor does not influence the distributions appreciably but it agrees with the total signals measured. A value of 1.2 usually decreases the average of the difference signal meaning that the signal deflected does not disappear outside the studied deflection range. Thus, it is possible to conclude how the signal is deflected within this range. The step size used for the pin collector displacement is equal to 0.63 mm. This is smaller than the width of the pin. In the figures the number of pin displacement steps is used since the center of the beam is not defined by the absolute pin position due to the slight variation of the laser focus position on the target between experiments.

#### Magnetic field at 0.10 T

The magnetic field strength of 0.10 T is given by two ferrite magnets of size 5×10×30 mm, one above and one below the beam. The time-pin position distributions for zero and negative collector bias have been measured for p(0) and D(0). In all four cases it is observed that the difference deflection distribution shows two different deflections. Two of the four cases are shown in Figs 15–18. The direct signal with no magnet demonstrates the symmetry of the beam flux. The largest bump in Figs 15 and 16 at approximately -2.5 steps is due to positive particles which are deflected from there to the valleys at 0 and +2–3 steps at total 2.5 and 5 steps (1.6 mm and 3.2 mm) from negative to positive lateral pin positions. It is directly seen that the deflected particles at 1.6 mm are slower than the other deflected particles. The values in Figs 17 and 18 are slightly different, with the bump at -2 steps and the minima at +0.5 and +3–4 steps. This means a total deflection of 2.5 and 5.5 steps, thus of 1.6 and 3.5 mm. See the Discussion section for further background for these choices of deflection distances. The total deflected signal in the range 0–50 ns as shown in the figures is relatively small, of the order of 25% from the peaks of the intensity distributions. This means that 75% of the signal is undeflected.

**Fig 15:** Signal time distributions at different lateral positions with no magnet (top) and with magnet (bottom). D(0) on the target, negative bias on pin collector, 0.10 T magnetic field strength.

**Fig 16:** Signal difference *I*(no magnet) - 1.2×*I*(magnet) from Fig 15. D(0) on the target, negative bias on pin collector, 0.10 T magnetic field strength. The difference signal shows positive particles on average being deflected from -2.5 steps to locations 0 and +2–3 steps, thus deflection of 2.5 and 5 steps.

**Fig 17:** Signal time distributions at different lateral positions with no magnet (top) and with magnet (bottom). p(0) on the target, zero bias on pin collector, 0.10 T magnetic field strength.

**Fig 18:** Signal difference *I*(no magnet) - 1.0×*I*(magnet) from Fig 17. p(0) on the target, zero bias on pin collector, 0.10 T magnetic field strength. The difference signal shows positive particles on average being deflected from -2 steps to locations 0 and +3–4 steps, thus deflection of 2.5 and 5.5 steps.

The particle mass can be calculated from the observed deflections. The particle velocity is higher than the apparent velocity from the time measurements, as shown above. This is due to the ejection of very fast particles from the decay of particles close to the target, with the time variation observed being due to particle formation and decay. Fig 19 shows the calculated result where the mass and velocity of the particles have been varied to give deflections of 1.6 and 3.5 mm, approximately equal to the observed deflections from the maximum to the minima in Figs15–18. The mass of the particles is definitely below unity, and the particles are thus mesons. Both kaons and pions are possible. Also muons are possible, at >500 MeV u^-1^ or >50 MeV.

**Fig 19:** Calculated particle mass and velocity giving deflections of 1.6 and 3.5 mm in an 0.10 T magnetic field. The particle energies used for the calculated points from left to right are 10, 20, 50, 100, 200, 500 MeV u^-1^ and 1 GeV u^-1^. The distances 1.6 and 3.5 mm correspond to 2.5 and 5.5 steps of the pin collector.

Further evidence exists in Fig 20, where the time distributions for the difference signal from Figs 15–18 are shown. The difference signals have approximately the same form as the direct signals, but some of the deflected parts of the signal are slower and some are faster, as indicated in the lower plot in Fig 20. If the 2.2 mm deflection is due to charged kaons, and the 3.5 mm deflection to pions, this would indicate that the pions have higher velocity than the kaons. Since the pions probably are formed by the decay of the kaons as in Eq. (5), their velocity may indeed be higher.

**Fig 20:** Difference signal time variation with the same data as in Figs 15–18. The deflected (minima) signal shows both a slow and a fast particle in one case (Fig 18). The theoretical curves give a decay time constant of 12–15 ns, thus indicating charged kaons.

In some experiments the decay time observed at the pin collector is shorter, down to 8 ns as in some distributions in Table 1. This indicates a lower velocity of the particles, which may decay before they reach the pin collector. This gives a signal shorter than the true decay time constant.

#### Magnetic field at 0.16 T

The magnetic field strength of 0.16 T is given by four ferrite magnets of size 5×10×30 mm, two on top of each other above and two likewise below the beam. The pin-collector position signal distributions for zero and negative collector bias have been measured for p(0) and D(0). Two of the four cases measured of the difference deflection distributions are shown in Figs.21–24, with the direct beam signal included in the figures to show the symmetry of the undeflected beam. Also the signal with the magnet in the beam is given for completeness. The difference distribution is single-peaked in the sideways deflection. The sign of the deflection agrees with positive particles and is in the range 4.0–5.0 steps, or 2.5–3.2 mm. Further details are given in the figure captions. The particle mass is calculated for deflections at 1.3 mm thus from the center and 3.2 mm with magnetic field strength of 0.16 T. These results are displayed in Fig 25 and show that the deflected signal is likely due to kaons or possibly pions. This conclusion is also correct if just the deflection from the center is considered due to the high velocity of the particles.

**Fig 21:** Signal time distributions at different lateral positions with no magnet (top) and with magnet (bottom). D(0) on the target, negative bias on pin collector, 0.16 T magnetic field strength.

**Fig 22:** Signal difference *I*(no magnet) - 1.2×*I*(magnet) from Fig 21. D(0) on the target, negative bias on pin collector, 0.16 T magnetic field strength. The difference signal shows positive particles being deflected from -2 or -2.5 steps to locations around +2 steps, thus around 4.0–4.5 steps.

**Fig 23:** Signal time distributions at different lateral positions with no magnet (top) and with magnet (bottom). p(0) on the target, negative bias on pin collector, 0.16 T magnetic field strength.

**Fig 24:** Signal difference *I*(no magnet) - 1.2×*I*(magnet) (bottom) from Fig 23. p(0) on the target, negative bias on pin collector, 0.16 T magnetic field strength. The difference signal shows positive particles being deflected from -2.5 steps to location around +2 steps, thus around 4.5 steps.

**Fig 25:** Calculated particle mass and velocity giving deflections of 1.3 and 3.2 mm in an 0.16 T magnetic field. The particle energies used for the calculated points from left to right are 10, 20, 50, 100, 200, 500 MeV u^-1^ and 1 GeV u^-1^. The distances 1.3 and 3.2 mm correspond to 2 and 5 steps of the pin collector.

The time distributions for the difference results in Figs 22 and 24 are shown in Fig 26, in the same way as the data in Fig 20 for Figs 16 and 18. The results agree well with decay of mainly charged kaons, with decay time of 12 ns. This means of course that the charged kaons may decay before they reach the deflecting magnetic field, forming pions and muons.

**Fig 26:** Difference signal time variation with the same data as in Figs 21–24. The theoretical curves give a decay time constant of 12 ns, thus for charged kaons.

### Neutral particles

Most particles in the magnet deflection experiments are not deflected appreciably. In the experiments, the fraction of particles not deflected is of the order of 75%, as noted above. In some cases, it is considerably higher. This means that they are either neutral (including photons) or so fast that they are not deflected in the magnetic field. Assuming that a deflection less than 0.63 mm (one lateral step for the pin collector) is not observable and thus can be counted as no deflection, the particle mass must be > 3 u at magnetic field 0.16 T to not be deflected at a velocity of 500 MeV u^-1^. Charged mesons will be deflected appreciably even at such a high velocity. Thus, it is concluded that most particles ejected are neutral. The time variation of this assumed neutral signal at the pin collector is not very informative. The apparent decay time is < 50 ns and thus caused by particles with intermediate velocities.

One possibility is of course that the neutral particles are ionizing photons, which interact with the collectors by ejecting photoelectrons and Compton electrons. Compton electrons can indeed be observed with positive bias on the collectors, as a peak at short time. However, most results do not agree with photons. The large difference between the signals at the inner and outer collectors means that photons cannot explain the signals. Such results are seen in Figs 5, 6, 7, 11 and 12 and summarized in Table 1. Most of these comparisons are for the entire signal, including the part of the signal identified to be due to charged particles. Stricter comparisons are possible for example using the data from experiments such as those in Figs 6 and 7 with magnetic deflection of the charged particles. In Figs 6 and 7, the magnets are used to deflect very fast charged particles, with a decay time constant of 13–16 ns, thus corresponding to fast charged kaons K^±^. Thus, the fastest particles are to a large part charged, not photons. Such results are also shown in Fig 27 both with D(0) and p(0) and with negative and zero collector bias. The signal to the outer collector is there shifted 3.2 ns to shorter time to compensate for the velocity of light between the collectors. It is clearly seen that the later parts of the curves are not identical, thus corresponding to particles with velocity somewhat less than the velocity of light. The first part of the curves represents particles moving at the velocity of light (photons or relativistic massive particles). Thus, the neutral signal is to a large part due to particles with a velocity somewhat less than the velocity of light. However, the distances to the two collectors have a ratio of 163/64 = 2.5 which would shift slower particles to much longer times if the particles did not change their velocity or mass during the flight between the collectors. This effect is shown by the recalculated signal curve in Fig 4.

**Fig 27:** Comparisons between signals at inner and outer collector, showing the signal not to be photons. The outer collector signal is shifted 3.2 ns to shorter times, corresponding to the time for light to move between the collectors. Thus particles moving close to velocity of light *c* and slower than *c* exist.

One possibility is that the neutral particles are of the H_*N*_(0) particle type, as suggested previously [16,17,21]. Such particles may be named quasi-neutrons, or quasi-dineutrons in the case of D_*N*_(0), and could remain neutral even after acceleration to very high velocities by the other fast ejected particles. However, their properties in this respect are not known. Another possibility is that the neutral particles are long-lived neutral kaons ${\text{K}}_{L}^{0}$ which have a decay time constant of 52 ns. This type of ${\text{K}}_{L}^{0}$ decay is shown in Fig 11. The most often observed time constant in the experiments is 13 ns, due to charged kaons K^±^. If similar numbers of neutral kaons and charged kaons are formed initially by the laser-induced nuclear processes, a large part of the neutral flux may be long-lived neutral kaons.

## Discussion

The time variation of the collector signals was initially assumed to be due to time-of-flight of the ejected particles from the target to the collectors. Even the relatively low particle velocity of 10–20 MeV u^-1^ found with this assumption [21–23] is not explainable as originating in ordinary nuclear fusion. The highest energy particles from normal D+D fusion are neutrons with 14.1 MeV and protons with 14.7 MeV [57]. The high-energy protons are only formed by the D + ^3^He reaction step, which is relatively unlikely and for example not observed in our laser-induced D+D fusion study in D(0) [14]. Any high-energy neutrons would not be observed in the present experiments. Thus, ordinary fusion D+D cannot give the observed particle velocities. Further, similar particle velocities are obtained also from the laser-induced processes in p(0) as seen in Figs 4, 6 and 7 etc, where no ordinary fusion process can take place. Thus, it is apparent that the particle energy observed is derived from other nuclear processes than ordinary fusion. It is clear that such laser-induced nuclear processes exist in p(0) as well as in D(0). The low laser intensity used here, of the order of 3×10^12^ W cm^-2^ makes it impossible to directly accelerate the particles (especially the neutral ones) to high energies. For example, in Refs. [58,59] more than 10^19^ W cm^-2^ was used to accelerate heavy ions to > 1 MeV u^-1^ energies, thus close to 10^7^ higher intensity than used here.

The experiments with two and three collectors made in this type of system [16,17,22,23] show more complex features. By comparing the different collector signals, it became clear that the time variation of the collector signals is not due to time-of-flight. Instead, it is obvious that the signal time variation is mainly due to time variation of the particle generation process at the laser target. This in turn implies that the particles move with much higher velocities than 10–20 MeV u^-1^ which was the apparent particle velocity. Different time variations of the signal at the collectors mean further that the same signal is not seen by two collector in-line, but that the particles in the beam are transformed during their flight between the collectors. Finally, the specific exponential decays observed in the time variations indicate clearly that several different decaying particles are generated at the laser target. The accurate modeling of the intermediate particle formation and decay used here means that the detailed behavior of the laser-induced processes can be investigated with confidence.

It could be thought that the signal time variation is due solely to processes on the target which vary with time. However, the different specific time variations of the signals at the two collectors in line contradict this. For example, in Figs 4 and 5 the signal variation at the inner collector is slower than at the outer collector. Thus the outer collector does not see the same signal, either due to different angular acceptance or due to decay of the particles in the beam. The dimensions of the collectors are in this case such that the same signal should be observed at both collectors in Fig 4. Thus, a real change of the particle flux is taking place between the collectors. In Figs 11 and 12 with model results collected in Table 1, it is clearly demonstrated that different signals are observed at the two collectors. It is thus concluded that the main signal variation is due to the time variation of the ejecting processes on the target with strong modifications due to decay processes during the transport in the beam.

If the process on the target which ejects the very fast particles was just a nuclear process with a decay time caused by energy loss from the high energy spot on the target, the apparent decay times would be quite arbitrary with no specific values found. This is not the case, but the time constants are reproducible and can also be measured accurately. One example is given in Fig 5, where the signal to the outer collector agrees accurately with the time constant 13 ns expected for charged kaon decay (12.4 ns at rest [51,55]). In Figs 13 and 14, the three main time constants are found with different laser pulse energies. Of course, in that case the time constants mix to some extent but no other time constant values are observed. This means that specific decay time constants are observed, and that the time variation of the signals is largely determined by such constants. From the decay time constants, it is clear that charged kaons are formed, which decay to charged pions and finally also to muons. The muons may not be easily detected by the metal collectors and have a long decay time constant of 2.2 μs which means that they may not decay appreciably before leaving the apparatus. When negative muons interact with materials by muon decay and capture, the time constant for the beta signal is of the order of a few μs. Thus, muon decay may not be directly observed here. The initial laser-induced processes on the target are not yet known, so it is here assumed that kaons and pions are formed more or less directly at the laser target from small H_*N*_(0) clusters, probably with *N* = 3–6. Direct evidence of the size of these clusters exists (to be published).

The charge of the mesons (kaons, pions) is observed to be positive by the magnetic deflection experiments. This means that they decay primarily to positive muons and finally positrons. The velocity of these particles will be quite high. Thus, processes like annihilation of the positrons will not exist close to the laser target since the positrons need to be thermalized before annihilation with electrons, and will not be easily detected in the experiments. One decay channel of low probability for positive kaons can also give negative pions and thus negative muons [51]. However, the detection of muons through muon decay and capture [3–5,60] with an example in Fig 3 (beta-like distribution) requires that negative muons are formed at quite large intensities. The possibility that seems to exist in the model used here is formation of negative muons by decay of neutral kaons ${\text{K}}_{L}^{0}$. These kaons interact relatively weakly with the collectors but they may as noted above constitute a large fraction of the neutral particles which pass undeflected by the magnets. The neutral kaons decay to give positive and negative pions and muons. The reason why they are not observed regularly from their decay lifetime here is that is it relatively long, at 52 ns. It is observed in one case in Table 1, and with 2 m collector distance from p(0) in Ref. [17]. It is also reported in Ref. [18]. The short-lived neutral kaon ${\text{K}}_{S}^{0}$ may give positive and negative pions directly [55].

The intermediate particle description agrees well with the results. This implies that the velocity of the particles is higher than the apparent particle TOF velocity of 10–20 MeV u^-1^. This velocity corresponds to a time from the target to the outer collector of 15 ns, or to 10 ns between the two collectors. It is shown here in Figs 6 and 7 that the fastest signal to the outer collector can be deflected by the magnet at the beam, which means that it is not due to photons. (Electrons are excluded as described above). Thus, these particles are relativistic at energies up to 0.75 *c* according to the direct time measurements between the two collectors. This corresponds to velocities higher than 500 MeV u^-1^. From the decay time and time between the two collectors for these relativistic particles, it was concluded that the particles are charged kaons with velocity of 280 MeV u^-1^ or kinetic energy of 150 MeV. A charged kaon may decay to a charged and a neutral pion. The excess energy in this process is 219 MeV, which means that very energetic particles are likely to be found also as decay products. They of course have a large probability to leave the beam.

The deflections of the particles in the magnetic fields observed are quite complex, as can be expected for a meson shower with several different meson types in the beam. For example, neutral, negative and positive kaons coexist in the beam, as concluded from the decay times observed. They decay in a complex fashion to pions and muons [51,55]. Even if the beam is symmetric without magnet as shown for example in Figs 21–24, this does not ascertain that also the different particle types have similar symmetric distributions in the beam. On the contrary, it must be expected that different types of particles have different spatial distributions in the beam, since they have different velocities from the complex particle decay patterns. One example may exist in Fig 16. If the beam was homogeneous, it would be expected that most of the signal flux was deflected by the magnetic field from the centerline of the beam. This is not the case, but the particles with larger transverse energies at the outer parts of the beam are the ones that are deflected most. Thus, it appears that neutral particles are more abundant in the center of the beam, or alternatively that the increase and decrease in particle number at the center are almost equal. This means that the deflections observed are from one side of the beam to the other, while the same type of particles from the other side of the beam leaves the beam. This is the reason for counting the deflections from the side of the beam to the other side, not only from the center. Both approaches are indeed included in the analysis in Figs 19 and 25.

The evidence from the calculations of the deflection in the magnetic fields in Figs 19 and 25 is clearly that the deflected particle masses are below unity. Mass 1 or 2 particles may explain the deflections only if they have relatively low velocity, at 10–20 MeV u^-1^ as initially thought to be the case but now shown not to be correct; the decay time constants cannot be explained as due to such particles. The signals at the outer collector do not agree at all with such slow particles. Comparing also to Fig 8 with the relativistic particle deflection means that mesons easily explain all these deflection results, and also the decay time constants. Thus the deflected particles in the magnetic fields are charged mesons, mainly with positive charge.

Another possibility could be that also negative mesons are formed and deflected by the magnetic fields. If negative mesons will give a negative current at the pin collector, the signal will not be so easily discriminated from the positive mesons giving a positive current with deflections of the same size but in the opposite direction. The difference signals in Figs 16, 18, 22 and 24 are in fact quite antisymmetric around the center, which could indicate similar negative and positive particle fluxes. The mechanism of charge ejection from the collectors for negative mesons should be the same as for positive particles, both giving a positive signal current, so the possibility of large negative meson fluxes cannot be supported.

The experiments using the small pin collector for TOF and magnetic deflection observe currents up to 1.2 mA, as seen in the figures. This means a peak current density of 25 mA cm^-2^ at the pin, or a factor of nine larger density of 200 mA cm^-2^ at the slit due to the difference of a factor of three in the distance to the laser spot. It is apparent that such a large current density is due to a very large number of emitted particles from the target.

It may thus be interesting to estimate the total energy released by the nuclear processes initiated by the laser. From Fig 6 the total signal at the outer collector is approximately 100 mV in 50 Ω resistance with negative bias, or a peak current of 2 mA. The total charge per laser pulse collected at 163 cm distance is thus approximately 3×10^−11^ As. Assuming an energy of the particles of 20 MeV gives 6×10^−4^ J per pulse. The fraction of the total sphere around the target covered by the outer collector is 6×10^−5^. An isotropic distribution over the whole sphere is likely since the direction of the beam to the collectors is quite arbitrary relative to the laser beam (45°) and the normal of the target (60°). This gives total particle energy of 10 J, much higher than the laser pulse energy of 0.2 J. In the experiment in Fig 6, an inner slit was in fact used with an opening of 6.6×10^−6^ of the total sphere, an even smaller value. This gives an energy of 90 J released, a factor 450 higher than the laser-pulse energy. Since the particle energy is higher than 20 MeV and the particles have velocities up to 200 MeV u^-1^, then the total energy released is correspondingly higher. The particles on average have mass less than unity but higher velocity than 20 MeV u^-1^, so a reasonable average for this estimate is 20 MeV. It should also be realized that the particles departing out from the beam on the way to the outer collector are not included, and they are probably the ones with the largest kinetic energy. Returning to Fig 6, the charged particles (deflected difference) have approximately a factor of 5 lower total intensity, thus corresponding to a total energy of 18 J per laser pulse in charged particles. These estimates of course depend on an assumed ejected isotropic distribution of particles around the laser interaction spot on the target. If it instead assumed that all the particles were ejected into a narrow cone of size 0.002 of the total sphere thus 2.4×10^−2^ sr (around 10° beam width) centered around the arbitrary direction towards the collectors, the energy released by the nuclear processes would be equal to the laser pulse-energy. Thus, it is safe to conclude that the nuclear processes in H(0) observed to give meson ejection release a large amount of energy.

## Conclusions

Mesons with different velocities are generated by the laser-induced nuclear processes in ultra-dense hydrogen D(0) and p(0). The highest velocities observed are in the range 0.6–0.75 *c*. Both charged kaons and pions are frequently observed from their decay time constants, while the neutral long-lived kaon ${\text{K}}_{L}^{0}$ with its longer decay-time is less frequently observed in the present experiments. It is probably observed as a long-lived foil-penetrating neutral particle, and it may be a large part of the neutral flux which is the main fast particle flux from the laser-induced nuclear processes. The magnetic deflection experiments give strong evidence for fast charged kaons and pions. Heavier or lighter particles cannot give the observed deflections.
